# Complexity and Entropy Analysis to Improve Gender Identification from Emotional-Based EEGs

**DOI:** 10.1155/2021/8537000

**Published:** 2021-09-21

**Authors:** Noor Kamal Al-Qazzaz, Mohannad K. Sabir, Sawal Hamid Bin Mohd Ali, Siti Anom Ahmad, Karl Grammer

**Affiliations:** ^1^Department of Biomedical Engineering, Al-Khwarizmi College of Engineering, University of Baghdad, Baghdad 47146, Iraq; ^2^Department of Electrical Electronic & Systems Engineering, Faculty of Engineering & Built Environment, Universiti Kebangsaan Malaysia, UKM, Bangi, Selangor 43600, Malaysia; ^3^Department of Electrical and Electronic Engineering, Faculty of Engineering, Universiti Putra Malaysia, UPM, Serdang, Selangor 43400, Malaysia; ^4^Malaysian Research Institute of Ageing (MyAgeing™), Universiti Putra Malaysia, Serdang, Selangor 43400, Malaysia; ^5^Department of Evolutionary Anthropology, University of Vienna, Althan Strasse 14, A-1090 Vienna, Vienna, Austria

## Abstract

Investigating gender differences based on emotional changes becomes essential to understand various human behaviors in our daily life. Ten students from the University of Vienna have been recruited by recording the electroencephalogram (EEG) dataset while watching four short emotional video clips (anger, happiness, sadness, and neutral) of audiovisual stimuli. In this study, conventional filter and wavelet (WT) denoising techniques were applied as a preprocessing stage and Hurst exponent (Hur) and amplitude-aware permutation entropy (AAPE) features were extracted from the EEG dataset. *k*-nearest neighbors (kNN) and support vector machine (SVM) classification techniques were considered for automatic gender recognition from emotional-based EEGs. The main novelty of this paper is twofold: first, to investigate Hur as a complexity feature and AAPE as an irregularity parameter for the emotional-based EEGs using two-way analysis of variance (ANOVA) and then integrating these features to propose a new CompEn hybrid feature fusion method towards developing the novel WT_CompEn gender recognition framework as a core for an automated gender recognition model to be sensitive for identifying gender roles in the brain-emotion relationship for females and males. The results illustrated the effectiveness of Hur and AAPE features as remarkable indices for investigating gender-based anger, sadness, happiness, and neutral emotional state. Moreover, the proposed WT_CompEn framework achieved significant enhancement in SVM classification accuracy of 100%, indicating that the novel WT_CompEn may offer a useful way for reliable enhancement of gender recognition of different emotional states. Therefore, the novel WT_CompEn framework is a crucial goal for improving the process of automatic gender recognition from emotional-based EEG signals allowing for more comprehensive insights to understand various gender differences and human behavior effects of an intervention on the brain.

## 1. Introduction

Perceiving gender based on human emotions has gained lots of research interest to investigate personal characteristics in neuroscience and psychology [1]. Gender differences primarily based on processing emotions have attracted precise interest due to their attainable utility in understanding human psychopathology such as depression and nervousness that might also be associated with the differential response of females and males to stress [2].

Thus far, few researchers have investigated gender variations primarily based on emotional changes [3], and most of them report substantial differences [2]. Accordingly, the kind of stimulus could be visual, auditory, or audiovisual stimuli. The visual stimuli and auditory stimuli are related to an increase or decrease in the sensorimotor rhythm amplitude [4]. To reveal personal characteristics that would be valuable in recognizing individual gender accurately in daily life, visual and auditory stimuli are considered as two common ways for human beings to elicit different emotional states [2]. Recently, researchers indicated that, to provide the best environment for automatic emotion recognition, they need to get the combined effect of both visual and auditory stimuli to elicit a specific emotional state [5]. Audiovisual elicitations utilizing short film video clips are usually used to elicit various conditions of emotion better compared to the other modalities [4, 6–9]. Hence, in this work, emotions were precipitated with the aid of the use of short audiovisual video clips.

From the psychological point of view, the emotional state can be distinguished and grouped into two emotional models: the discrete model and the dimensional model. The discrete model comprises a lot of discrete emotional states that are identified to be one of the core emotions, and all other different emotions are considered part of these primary emotions (anger, fear, disgust, surprise, happiness, and sadness) or an aggregate of them [10, 11]. The dimensional model is a two-dimensional (2D) cognitive-emotional state model that is broadly utilized in mapping emotion recognition applications. It plots emotions on two scales, valence-arousal plots, where valence is in the horizontal axis and is considered as the polarity or the quality of an emotion ranging from unpleasant to pleasant and arousal is in the vertical axis and is considered as the intensity of emotion ranging from calm to excited [12]. Therefore, the 2D cognitive-emotional state model is the mapping of all emotions onto the valence-arousal graph, as portrayed in the circumplex model of emotion [13, 14]. Other researchers have proposed a three-dimensional (3D) cognitive-emotional state model which takes into consideration the attention-rejection property in addition to the 2D model [8, 15–17].

In this study, the conventional filter and wavelet (WT) denoising techniques were applied as a preprocessing stage to the EEG dataset. Hurst exponent (Hur) complexity feature and amplitude-aware permutation entropy (AAPE) irregularity parameter have been computed to investigate the gender changes of the emotional-based EEGs. Subsequently, the individual performances of these features were statistically examined using two-way analysis of variance (ANOVA) to recognize a gender-specific role in the brain-emotion relationship for females and males during four short emotional video clips (anger, happiness, sadness, and neutral) of audiovisual stimuli. Then, the used features were combined as a novel complexity and irregularity features (CompEn) hybrid feature fusion set towards developing the novel WT_CompEn framework for automated gender recognition system on EEG for gender identification. Finally, kNN and SVM classification techniques were used for automatic gender identification of emotional-based EEG datasets. The performances of these classifiers were examined on Hur and AAPE individually and on the CompEn feature set.

To the best of author's knowledge, the contribution of a gender-precise role in the brain-emotion relationship has been tended to in this work. Therefore, the main novelty of this paper is threefold. First, it aims to propose an automated gender recognition system based on EEG data of different emotional states acquired using low-cost wireless EEG devices. This can be done by investigating the changes in complexity and irregularity features of the emotional-based EEGs using statistical analysis. Then, integrate the employed features as CompEn feature set towards developing the novel WT_CompEn framework as a core for automated gender recognition system feature set to be sensitive for identifying gender differences of emotional-based EEG signals. Third, the EEG elicitation convention and the EEG estimation system are utilized without precedent for this investigation for emotion data obtaining, and that may make gender contrast more articulated and may accomplish better performance.

## 2. Related Works

Over the last decade, studies have indicated that the possible adequacy of biomedical signs for recognizing people by exploring gender differences based on emotional changes would be elicited using different physiological measurements such as electrocardiogram (ECG) [18] and electroencephalogram (EEG) [6, 19]. Several studies illustrated the gender differences and classification from ECG signal analysis [20, 21], while in other studies, the gender has been classified based on using EEG signals [22, 23].

Characterized by wide availability, affordability, and lack of invasiveness, EEG is a clinical instrument capable of monitoring data processing in millisecond accuracy with a high level of temporal resolution [24], Therefore, it has neurophysiology applications for the detection and differentiation of modifications in the brain [24, 25].

A wide range of brain disorders, including seizures, attention-deficit hyperactivity disorder (ADHD), and Alzheimer's disease (AD)/vascular dementia (VaD), have been detected based on EEG signals, while mental tasks and sleep stages have been classified based on such signals as well [23–26]. The latest research has employed EEG for high time-resolution evaluation of affective moods in people [26–29]. Recently, EEG has been generally utilized to assess human emotional states with high time resolution [6, 30, 31]. Given the important insight that it can provide in this regard, EEG may be a promising biomarker for the appraisal of different affective reactions from an EEG dataset with multiple channels across brain regions [32]. To give an example of such research, brain waveforms were used in [33] to develop a method of uninterrupted music emotion detection. Similarly, in [34], real-time techniques of human emotion detection based on EEG were employed to devise an integrated music therapy for the identification of present affective moods according to neurofeedback and patient-specific customization of treatment.

Besides being highly informative about brain physiology, EEG signals could potentially be biomarkers of brain linear and nonlinear behavior [26, 27, 35–37]. The Hurst exponent (Hur) [6, 38] and fractal dimension (FD) [39, 40] are among the nonlinear techniques that have been adopted for the representation of complex affective tasks and for the examination of complicated dynamic data generated by the brain cortex [33, 41].

EEG signals are considered dynamic systems lacking stability, and the uncertainty of such systems can be determined by employing the nonlinear parametric index of entropy [42]. Research into cognitive mental states, sleep states, and approaches for categorizing affective levels has benefitted from the application of entropy to EEG signals [35, 43–45]. Furthermore, the use of a range of entropies for the identification of biological gender based on EEG could be useful in clinical analyses, especially on social emotion, individual identification, response to therapy, clinical effectiveness, and side effects [46]. To give an example, in [1], human emotions triggered by video clips were examined based on sample entropy (SampEn), approximate entropy (ApEn), and permutation entropy (PerEn), as these entropies are resistant to noise and can effectively measure time series complexity. In a different study, the analysis of EEG signals for clinical evaluation was conducted based on PerEn entropy and symbolic transfer entropy, hinting at the relational ability of the employed EEG entropy examination with clinical cases of different cognitive conditions [47]. Another type of entropy suggested for EEG examination is fuzzy entropy (FuzEn), involving the substitution of Heaviside functions with fuzzy membership functions [48, 49]. According to existing studies, the issue of entropy mutation is mitigated by FuzEn, but on the downside, the relevant information is lost when employing such entropy techniques because they entail single-scale analysis. Whereas the speed of SampEn is better compared to FuzEn, greater consistency and reduced reliance on data length are demonstrated by FuzEn [50]. ApEn [51], SampEn [52], FuzEn [53], and PerEn [54] constitute the four most popular entropy predictors within the context of EEG signal processing [50]. To identify how affective-based EEG signals across the brain differ between genders, the present work concentrates on EEG-derived indices.

Support vector networks (SVNs), artificial neural networks (ANNs), *k*-nearest neighbors (kNN) and support vector machine (SVM) classifiers [55], and hidden Markov models (HMM) have all been employed to investigate automatic algorithms for a system of gender categorization [56, 57]. For instance, the SVM classifier was used in [22] to devise an EEG signal-based automatic system of age and gender detection, while EEG data related to resting state were the basis of a model of automatic gender detection in [1]. In other research, EEG sensors with wavelet transform frequency breakdown for feature extraction and random forest classifier enabled the creation of an automatic system for detecting age and gender in resting state with eyes closed [58, 59].

Most gender detection studies using EEG signals based on emotional response focused on the linear analysis using spectral relative powers [30, 60, 61]. However, other researchers have used nonlinear features to investigate brain complexity [62–64]. In the current study, we aim to understand the role of EEG for gender identification using the integrated entropy and spatial features to characterize the emotional-based signals by examining different brain region behaviors during audiovisual video clips. Integrated features are essential for an automatic gender detection system to perform effectively and be solidly reliable. In this context, the impact of gender discrepancies on the elements of EEG-based systems of affective reaction detection and the general performance of such systems are worth investigating. To this end, computation of entropy features was done to highlight the gender variability occurring in affective-based EEG systems.

## 3. Materials and Methods

Figure 1 illustrates the block diagram of the proposed study.

### 3.1. EEG Acquisition and Recording

A mobile and affordable Emotiv EPOC EEG 14-channel headset (Emotiv Systems, Inc., San Francisco, CA) was employed in this work to capture EEG signals labeled as AF3, F7, F3, FC5, T7, P7, O1, O2, P8, T8, FC6, F4, F8, and AF4, with the common mode sense (CMS) left mastoid and the driven right leg (DRL) being referenced as ground. The positioning of the sponge-based electrodes used by the headset was done according to the 10–20 system, while a band-pass filter of 0.5–70 Hz frequency facilitated the filtering of electrode data. The frequency of sampling was 128 Hz, with 0.51 mV resolution.

The study recruited a total of ten participants (6 males and 4 females; the age of 22.6 ± 2.75 years, mean ± standard deviation (SD)), all university students, aged between 18 and 24 years. Before beginning the research, each participant underwent an evaluation to ensure no prior history of neurological or psychiatric issues and was then presented with an informed consent form (ICF) which they were requested to sign before participating in the study.

During the EEG recording procedure, subjects were asked to remain relaxed and calm for the entire EEG recording duration to minimize the data reading artifacts resulting from movements. The evaluation of the 3 emotion states (anger, sadness, and happiness) along with the neutral condition was conducted by allowing the participants to view various short emotionally stimulating video clips, with audio, following which the participants were allowed some time to evaluate and grade their responses to the clips employing a self-assessment questionnaire, followed by a break of 45 seconds before viewing the next video clip (Figure 2) [65].

The running time of the various video clips varied from one to the other, with the longest having a duration of four minutes. The emotional video clips used were selected based on those recommended by Rottenberg et al. [65]. As previously mentioned, participants were asked to evaluate the strength of their emotional response to each clip using a five-point-scale SAQ; participants were asked to select either 1 (very low), 2 (low), 3 (medium), 4 (high) or 5 (very high) to evaluate the degree of emotion experienced [31].

To enable the participants to view the affective video clips, the used video clips were in German language and the virtual emotion presenter (VEP) software from the University of Vienna was employed. This software was chosen because it not only permits arbitrary viewing but also documents extra sources of data. The experimental work was conducted in the Anthropology Research Laboratory, and besides the VEP software, the equipment used included the regular laboratory ambient lighting, LCD for screening the video clips, and stereo speakers so that the video clips could be accompanied by uninterrupted sound at a level acceptable to the participants (Figure 3). The Helsinki declaration and subsequent refinements were followed in every research procedure.

### 3.2. Preprocessing Stage

Since most artifacts occurring in EEG signals were overlapping with brain activity, preprocessing is essential in EEG signal processing.

#### 3.2.1. Conventional Filtering

In this context, conventional filters were used as an initial stage to process each channel of the recorded EEG datasets. A notch filter at 50 Hz was used to remove the power line interference noise [32], and a fourth-order Butterworth bandpass filter was applied with a 0.5–64 Hz frequency range to limit the band of the recorded EEG signals [66].

#### 3.2.2. Wavelet Analysis

WT has the ability in resolving EEG into specific time and frequency components by providing a good time resolution and poor frequency resolution at high frequencies and good frequency resolution and poor time resolution at low frequencies. The DWT is a fast nonredundant transform used in practice for analyzing both the low- and high-frequency components in the EEG signals because it requires less computational time than the continuous WT (CWT) [67]. The DWT can be processed by obtaining the discrete value of the parameters *a* and b, as in equation (1). It can be obtained as a set of decomposition functions of the correlation between the signal *f*(*t*) and the shifting and dilating of one specific function called mother wavelet function *ψ*(*t*). MWT is shifted by the location parameter (*b*) and dilated or contracted by frequency scaling parameter *a*, as in the following equation [8, 16, 17, 36, 68–70]:

(1) $$\begin{array}{c} {\text{DWT}}_{m,n}\left(f\right)=a_{0}^{-\left(m/2\right)}\int f\left(t\right)\psi \left(a_{0}^{-m}t-nb_{0}\right)\text{d}t, \end{array}$$

where *a*_0_ and *b*_0_ values are set to 2 and 1, respectively.

(2) $$\begin{array}{c} \psi_{a,b}\left(t\right)=\frac{1}{\sqrt{a}}\psi \left(\frac{t-b}{a}\right),\;a\in {\mathbb{R}}^{+},\;b\in \mathbb{R}. \end{array}$$

SURE threshold is an adaptive soft thresholding method, which aims to determine the threshold limit for each level based on Stein's unbiased risk estimation [71] and commonly used value in [72–74].

In this study, the sampling frequency was 128 Hz and the EEG dataset was subjected to “sym9” from the Symlets family with a four-decomposition level of five subband EEG signals. Among the five subbands, cD1, cD2, cD3, and cD4 represented the decomposition detail coefficients and cA is the decomposition approximation coefficient. The SURE threshold is an adaptive soft thresholding method that is used to find the threshold limit for each level based on Stein's unbiased risk estimation [70, 74].

### 3.3. Features Extraction Stage

Because of the complicated structure of the brain and its ability to perform multiple and complex sophisticated cognitive tasks, the brain neurons are considered to be governed by nonlinear dynamic phenomena. EEG signals have been used to investigate the chaotic behavior of the brain from nonlinear time series [75, 76]. Since the EEG spectral-band analysis was unable to illustrate the electrical activity of the brain and the underlying mechanisms of the brain function, the nonlinear analysis based on dynamics information needs to be investigated. The present study was undertaken to examine the gender differences from emotional-based EEG background activity with two different features: Hurst exponent (Hur) and amplitude-aware permutation entropy (AAPE) to illustrate the complexity and irregularity features in detecting gender differences [63, 77–79]. Indeed, the used features were selected based on previous studies due to their usefulness and effectiveness in discriminating the EEG signals [35, 80, 81]. In this stage, the filtered EEG datasets were segmented into 3 trials, and each trial includes 10 seconds of each video clip viewed (3 × 10 second period) with 1280 data points.

#### 3.3.1. Hurst Exponent (Hur)

Hur is a measure that has been widely used to evaluate the self-similarity and correlation properties of fractional Brownian noise and the time series produced by a fractional (fractal) Gaussian process. Hur is used to evaluate the presence or absence of long-range dependence and its degree in a time series. However, local trends (nonstationarities) are often present in physiological data and may compromise the ability of some methods to measure self-similarity. Hur is the measure of the smoothness of a fractal time series based on the asymptotic behavior of the rescaled range of the process. In time series analysis of EEG, Hur is used by [38, 80] to characterize the nonstationary behavior of the EEG signals. Hur is defined as

(3) $$\begin{array}{c} \text{Hur}=\frac{\log\left(R/S\right)}{\log\left(T\right)}, \end{array}$$

where *T* is the duration of the sample of data and *R*/*S* is the corresponding value of the rescaled range. The above expression is obtained from Hurst's generalized equation of time series that is also valid for Brownian motion [82].

#### 3.3.2. Amplitude-Aware Permutation Entropy (AAPE)

AAPE has been proposed to consider the amplitude information from permutation entropy (PE) to overcoming the PE shortcoming of considering the order of the amplitude and discarding the information regarding the amplitude, besides the equal amplitude values in each embedded vector are not considered.

To estimate AAPE, assume *y*={*y*_*t*+(*j*_1_ − 1)*l*_,  *y*_*t*+(*j*_2_ − 1)*l*_,…, *y*_*t*+(*j*_*d*_ − 1)*l*_} is the time series, where *j* is the time index of the element in the reconstruction vector, a vector including the *d*! potential symbol patterns of *π* motifs, where *d* is the embedded dimension, which determines how much information is contained in each vector, and *l* is the time delay of the order pattern *i*, *i*=1,2,…, *d*!. To calculate AAPE, for each *π*_*i*_, *p*(*π*_*k*_) demonstrates the relative frequency as follows [81]:

(4) $$\begin{array}{c} p\left(\pi_{k}\right)=\left\{\begin{array}{cc} p\left(\pi_{i}^{d,l}\right)+\left[A/d\sum_{k=1}^{d}\left|x_{i+\left(k-1\right)l}\right|+1-A/d-1\sum_{k=2}^{d}\left|x_{i+\left(k-1\right)l}-x_{i+\left(k-2\right)l}\right|\right] & \text{if }p\left(\pi_{i}^{d,l}\right)=0\\ \frac{p\left(\pi_{i}^{d,l}\right)}{\sum_{i=1}^{N-d+1}\left[A/d\sum_{k=1}^{d}\left|x_{i+\left(k-1\right)l}\right|+1-A/d-1\sum_{k=2}^{d}\left|x_{i+\left(k-1\right)l}-x_{i+\left(k-2\right)l}\right|\right]} & \text{otherwise} \end{array}\right\},\\ \text{AAPE}\left(d,l,n\right)=-\sum_{\pi_{k}=1}^{\pi_{k}=dl}p\left(\pi_{k}\right)\ln\;p\left(\pi_{k}\right). \end{array}$$

When all motifs have equal probability, the largest value of AAPE is obtained at *l*=1. For 30 seconds, *N*=3840 samples, 3 windows of 10-second length (1280 samples) were extracted from the original EEG time series for each 14 channels.

#### 3.3.3. Complexity and Entropy Features Fusion

To get an efficient gender recognition model in terms of high accuracy recognition rates and to have more insights on the mental processes for females and males, the Hur index of complexity and AAPE index of irregularity have been combined to develop a new hybrid index of complexity-entropy (CompEn) set of feature.

### 3.4. Statistical Analysis Stage

This study intends to investigate the significance of Hur and AAPE features to be reliable indices in detecting gender differences in anger, happiness, sadness, and neutral emotional states. Therefore, statistical analysis has been conducted using SPSS statistical tool version 22. Two sessions of two-way analyses of variance (ANOVA) were performed to realize the significant differences among the emotions (i.e., anger, happiness, sadness, and neutral), and Hur was considered for the first session and AAPE was considered for the second session. Hur and AAPE were applied as dependent variables. The group factor (i.e., female and male) was the independent variable. The significance was set at *p* < 0.05. Moreover, the study was aimed to test the hypothesis that the gender differences from emotional-based EEG performed from the complexity and entropy-based features would be different between females and males.

## 4. Classification Stage and Performance Measures

The last stage for identifying neurophysiological changes in females and males is using the classification model. In this study, *k*-nearest neighbors (*kNN*) and support vector machine (SVM) were used.

Given that the majority of the learning algorithms assume a balanced class distribution, their results typically favor the predominant class that gives poor class predictions. The class imbalance in the dataset highly affects the quality of the classification model. However, given that the minority class cannot be easily discriminated against, the classifier can simply classify each instance as the majority class. In this study, the minority class was represented by the females. A synthetic oversampling technique (SMOTE) was applied to overcome the data imbalance [83]. The classifier parameters and percentage of oversampling were determined via 10-fold cross-validation using a grid search approach to avoid overfitting and bias in the classification analysis [84]. The available dataset was divided into 10 equal size disjoint subsets. One of these subsets was used as the test set, while the remaining nine subsets were combined into a training set to learn the classifier. This procedure was performed 10 times, which resulted in 10 accuracies. The average of these accuracies represented the 10-fold cross-validation accuracy of learning from this dataset [85]. Given that SMOTE changes the dataset, the percentage of oversampling were combined with the parameters. Therefore, those parameters that are found with different SMOTE percentages may not be the same. Using only the training set, the SMOTE was used to equalize the frequency of the classes [86, 87].

kNN is one of the most popular nonparametric classification algorithms, it is more robust when *k* > 1 particularly to reduce the influenced noisy points within the training set. In this study, the Euclidean distance was utilized as a similarity measure to classify each trial by kNN. The classifier was trained to obtain the best value of *k*=7 that maximizes the overall classification performance evaluation. kNN with 7 neighbors classifiers were selected based on previous work [9, 28, 29, 43, 77, 79, 88].

Optimization of the complexity parameter *C* with a range of −4 ≤ log_10_(*C*) ≤ 4 in *C* values *C* ∈ {0.0001, 0.001, 0.01, 0.1, 0,10,100,1000,10000} on the training set via ten-fold cross-validation yielded ideal outcomes for the SVM classifier. During testing, *C* corresponding to 10 gave optimal results for *C* values. The multiclass SVM classifiers were applied based on the radial basis function (RBF) kernel. Furthermore, the training dataset was used to determine the minimum misclassification rate, which in turn helped to obtain the smoothing parameter *σ* in the context of SVM training. Methodical variation of *σ* value in different training episodes is the only way of determining the ideal *σ*. Hence, in this work, variation of the *σ* value was done in the range of 0.1–1 at 0.1 intervals. A *σ* value of 0.5 was established to be associated with the minimum misclassification rate.

The performance of the proposed framework was evaluated using the values of average classification accuracy, confusion matrix, receiver operating characteristic curve (ROC), and area under the curve (AUC).

## 5. Results and Discussions

### 5.1. Results of Preprocessing Stage

As previously described, the EEG signal datasets were filtered by conventional filters and subjected to the WT denoising technique.  Figure 4 illustrates the data obtained from channel 7, representing the frontal brain area when subjected to the emotional state of anger. Observation shows that the artifactual signal elements (blue lines) present in the raw EEG signal were successfully blocked during signal denoising, resulting in the clean EEG signal (red line).

### 5.2. Results of Statistical Analysis

The statistical characterization of the differences in Hur and AAPE females and males will be discussed in the following sections.

#### 5.2.1. Results of Hurst Exponent (Hur)

The boxplots of Figure 5 indicate the overall pattern of Hur feature response for the two group factor distribution (i.e., female and male) from emotional-based EEG signals. It can be observed that Hur provides a significant variation with a useful way to visualize the characteristics of responses for the female and male group factors. Furthermore, boxplot analysis demonstrates the median value, as the value inside the boxplots is the median value of the distribution. The typical boxplot has lines at the upper median and lower quartile values. Figure 5 confirms the suitability of the feature for pattern classification.

Moreover, to recognize the importance of the complexity feature Hur method for the pattern classification, statistical analysis using two-way ANOVA was conducted on the Hur features. In this analysis, the group factor (i.e., female and male) was the independent variable, whereas the Hur features were the dependent variable. The significance for all statistical tests was set at *p* < 0.05. Normality was then assessed using the Kolmogorov–Smirnov test, whereas homoscedasticity was verified using Levene's test. The post hoc comparison was performed through Duncan's test.

Figure 6 illustrates the comparative plot of Hur which was estimated to discriminate between females and males based on anger, happiness, sadness, and neutral emotional states based on EEG signal complexity. Anger, happiness, and neutral were statistically significant from sadness, particularly for females, whereas anger, happiness, and sadness were statistically significant from neutral for males. One can see that the females had significantly lower Hur values at the four different emotional states compared to males ((Hur_anger,happiness,sadness,neutral _(Females) < Hur_anger,happiness,sadness,neutral _(Males))) with significant differences (*p* < 0.05). These results suggest that the EEG activities of females are significantly less complex for males.

#### 5.2.2. Results of Amplitude-Aware Permutation Entropy (AAPE)

The boxplots of Figure 7 indicate the overall pattern of AAPE feature response for the two group factor distribution (i.e., female and male) from emotional-based EEG signals. It can be observed that AAPE provides a significant variation with a useful way to visualize the characteristics of responses for the female and male group factors. Furthermore, boxplot analysis demonstrates the median value, as the value inside the boxplots is the median value of the distribution. The typical boxplot has lines at the upper median and lower quartile values. Figure 7 confirms the suitability of the feature for pattern classification.

Moreover, to recognize the importance of the complexity feature AAPE method for the pattern classification, statistical analysis using two-way ANOVA was conducted on the AAPE features. In this analysis, the group factor (i.e., female and male) was the independent variable, whereas the AAPE features were the dependent variable. The significance for all statistical tests was set at *p* < 0.05. Normality was then assessed using the Kolmogorov–Smirnov test, whereas homoscedasticity was verified using Levene's test. The post hoc comparison was performed through Duncan's test.

In this study, AAPE has been used for discriminating females from males based on anger, happiness, sadness, and neutral emotional states based on EEG signal irregularities.  Figure 8 illustrates the comparative plot of AAPE; it can be observed that sadness was statistically significant from neutral anger and happiness. Notably, EEG significantly had lower AAPE values in happiness and sadness for females compared to males (AAPE_happiness,sadness_(Females) < AAPE_happiness,sadness_(Males)), whereas the females had higher AAPE values for anger and neutral emotional states compared to males (AAPE_anger,neutral _(Females) < AAPE_anger,neutral _(Males))(*p* < 0.05). These results suggest that EEG had regular behavioral activities for both females and males.

### 5.3. Results of Classification Stage

This study has dealt with emotional-based EEG signals for gender identification problems. The key design decisions for kNN and SVM used in the classification are the training process, as they depend on the size of the training set and the test set. However, to comparatively evaluate the performance of the proposed classifiers, the classifiers employed in this work were trained on the same training data set and tested on the testing data set.

#### 5.3.1. Results of Hurst Exponent and Classification Performance

Tables 1 and 2 display the confusion matrix for female and male identification from emotional-based EEG signals using Hur complexity index with kNN and SVM classifiers, respectively, in which correct recognition is shown on the diagonal and substitution errors are off-diagonal.

In Table 1, the two diagonal cells show the percentage of correct classification using kNN classifier. For example, females are correctly classified with 58.3%; similarly, 100% are correctly classified as males, whereas 41.7% of females are incorrectly classified as males.

The results show that kNN classifier can differentiate females and males from emotional-based EEG signals with a high accuracy of 83%. Moreover, Figure 9 illustrates the ROC curve and the AUC value obtained from the investigation of the Hur features.

In Table 2, the two diagonal cells show the percentage of correct classification using SVM classifier. For example, females are correctly classified with 80%; similarly, 90% are correctly classified as males. Moreover, 20% of females are incorrectly classified as males, whereas 10% of males are incorrectly classified as females.

The results show that SVM classifier can differentiate females and males from emotional-based EEG signals with a high accuracy of 86.7%. Moreover, Figure 10 illustrates the ROC curve and the AUC value obtained from the investigation of the Hur features.

#### 5.3.2. Results of Amplitude-Aware Permutation Entropy and Classification Performance

Tables 3 and 4 display the confusion matrix for female and male identification from emotional-based EEG signals using AAPE entropy index with kNN and SVM classifiers, respectively, in which correct recognition is shown on the diagonal and substitution errors are off-diagonal.

In Table 3, the two diagonal cells show the percentage of correct classification using kNN classifier. For example, females are correctly classified with 100%; similarly, 77.8% are correctly classified as males, whereas 22.2% of males are incorrectly classified as females.

The results show that kNN classifier can differentiate females and males from emotional-based EEG signals with a high accuracy of 86.7%. Moreover, Figure 11 shows the ROC curve and the AUC value obtained from the investigation of the AAPE features.

In Table 4, the two diagonal cells show the percentage of correct classification using the SVM classifier. For example, females are correctly classified with 90%; similarly, 90% are correctly classified as males. Moreover, 10% of females are incorrectly classified as males, whereas 10% of males are incorrectly classified as females.

The results show that the SVM classifier can differentiate females and males from emotional-based EEG signals with a high accuracy of 90%. Moreover, Figure 12 shows the ROC curve and the AUC value obtained from the investigation of the AAPE features.

#### 5.3.3. Results of CompEn Hybrid Index and Classification Performance

Tables 5and 6 display the confusion matrix for female and male identification from emotional-based EEG signals using CompEn hybrid index with kNN and SVM classifiers, respectively, in which correct recognition is shown on the diagonal and substitution errors are off-diagonal.

From Table 5, the two diagonal cells show the percentage of correct classification using kNN classifier. The females are correctly classified with 91.7%; similarly, 100% are correctly classified as males, whereas 8.3% of males are incorrectly classified as females.

The results show that females can be differentiated with a high accuracy of 96.7% using kNN classifier to discriminate females and males from emotional-based EEG signals. Moreover, Figure 13 illustrates the ROC curve and the AUC obtained from the investigation of the CompEn features; the AUC was 0.96 and indicates that the proposed CompEn hybrid index exhibits robust classification performance in discriminating females and males from emotional-based EEGs.

In Table 6, the two diagonal cells show the percentage of correct classification using the SVM classifier. For example, females are correctly classified with 100%; similarly, 100% are correctly classified as males.

The results show that females can be differentiated with a high accuracy of 100% using SVM classifier as a benchmark technique to discriminate females and males from emotional-based EEG signals. Moreover, Figure 14 illustrates the ROC curve and the AUC obtained from the investigation of the CompEn features; the AUC was 1 and indicates that the proposed CompEn hybrid index exhibits robust classification performance in discriminating females and males from emotional-based EEGs.

Therefore, the results showed that the proposed WT_CompEn framework significantly increases the classification accuracy. Indeed, the results emphasize the crucial role played by the novel proposed WT_CompEn framework in the EEG signal processing chain, particularly in the classification results.

Gender recognition framework using emotional-based EEG signals has been performed under MATLAB R2021a on a laptop with processor Intel Core i7-8550U CPU @ 1.80 GHz and 1.99 GHz using 16.0 GB RAM and 64-bit operating system.

However, some limitations also need to be considered in this study; for instance, the sample size was small and an additional analysis with a large database should be performed in the future. Despite this, the different attributes of offline and online categorizations call for additional investigations based on real-time online experiments to validate the results obtained. Such limitations notwithstanding, there is an agreement between the results reported by this work and those of other studies, which confirmed the ability of EEG signals to identify the most gender discrepancies regarding anger, sadness, happiness, and neutral emotions and those discrepancies were reflected in the EEG bands as well [8, 17, 63, 77–79].

## 6. Conclusion

Conventional filters and WT techniques were used in the preprocessing stage to denoise the EEG datasets of 10 subjects while watching four short emotional video clips (anger, happiness, sadness, and neutral) of audiovisual stimuli. In the second stage, Hur complexity feature and AAPE irregularity parameter have been computed to investigate the gender changes of the emotional-based EEGs. Moreover, ANOVA has been used to statistically examine the individual performance of the used features to recognize a gender-specific role in the brain-emotion relationship for females and males during four short emotional video clips. Then, the used features were combined as novel complexity and irregularity features CompEn hybrid feature set towards developing the novel WT_CompEn framework as a core for an automated gender recognition system on EEG for gender identification. Finally, kNN and SVM classification techniques have been used for automatic gender identification of emotional-based EEG datasets. The performances of these classifiers were examined on Hur and AAPE individually and on the CompEn hybrid feature set. Potentially, the novel WT_CompEn framework can be used to identify gender differences from emotional-based EEG signals with high classification results.

This study has a primary limitation of the small sample size examined during the experiment. Therefore, further investigations will be carried out on a larger database in the future. Like every work, this study has advantages and weak points. However, gender detection has many advantages as well as applications such as health care, human-computer based interaction, knowing consumer preferences for online retailers, and biometric. Our findings approve the effectiveness of using complexity and irregularity features and CompEn hybrid feature set towards developing the novel WT_CompEn framework as an automated gender recognition system on EEG for gender identification. This study reveals useful insights about gender detection from emotion-based EEG classification. More investigation can be performed to describe the physiological meaning of the extracted features. Other classification approaches can be employed in further studies. In the future, researchers can decrease the computation cost and processing time. It is worth mentioning that the advantages of the current study outweigh the drawbacks.

## Figures and Tables

**Figure 1:** The block diagram of the proposed study.

**Figure 2:** The experimental protocol of emotion [9].

**Figure 3:** Setup of the experimental room with presentation TV and the recorders.

**Figure 4:** The denoising results after preprocessing stage for channel F7.

**Figure 5:** Boxplots for the Hur feature extraction method for gender distribution from emotional-based EEG signals. The dark black line represents the median values.

**Figure 6:** Comparative plot of the four tested emotional states for females and males using Hurst exponent complexity feature.

**Figure 7:** Boxplots for the AAPE feature extraction method for gender distribution from emotional-based EEG signals. The dark black line represents the median values.

**Figure 8:** Comparative plot of the four tested emotional states for females and males using amplitude-aware permutation entropy feature.

**Figure 9:** ROC curve and the AUC values of gender classification from emotional-based EEGs using Hurst exponent features and kNN classifier.

**Figure 10:** ROC curve and the AUC values of gender classification from emotional-based EEGs using Hurst exponent features and SVM classifier.

**Figure 11:** ROC curve and the AUC values of gender classification from emotional-based EEGs using amplitude-aware permutation entropy and kNN classifier.

**Figure 12:** ROC curve and the AUC values of gender classification from emotional-based EEGs using amplitude-aware permutation entropy and SVM classifier.

**Figure 13:** ROC curve and the AUC values of gender classification from emotional-based EEGs using proposed CompEn hybrid features and kNN classifier.

**Figure 14:** ROC curve and the AUC values of gender classification from emotional-based EEGs using proposed CompEn hybrid features using SVM classifier.

**Table 1:** Confusion matrix calculations for gender classification from emotional-based EEGs using Hurst exponents and kNN classifier.

Predicted	Actual		
	Gender	Females (%)	Males (%)
Hur	Females	58.3	41.7
	Males	0	100

**Table 2:** Confusion matrix calculations for gender classification from emotional-based EEGs using Hurst exponents and SVM classifier.

Predicted	Actual		
	Gender	Females (%)	Males (%)
Hur	Females	80	20
	Males	10	90

**Table 3:** Confusion matrix calculations for gender classification from emotional-based EEGs using amplitude-aware permutation entropy and kNN classifier.

Predicted	Actual		
	Gender	Females (%)	Males (%)
AAPE	Females	100	0
	Males	22.2	77.8

**Table 4:** Confusion matrix calculations for gender classification from emotional-based EEGs using amplitude-aware permutation entropy and SVM classifier.

Predicted	Actual		
	Gender	Females (%)	Males (%)
AAPE	Females	90	10
	Males	10	90

**Table 5:** Confusion matrix calculations for gender classification from emotional-based EEGs using CompEn hybrid fusion index and kNN classifier.

Predicted	Actual		
	Gender	Females (%)	Males (%)
CompEn	Females	91.7	8.3
	Males	0	100

**Table 6:** Confusion matrix calculations for gender classification from emotional-based EEGs using amplitude-aware permutation entropy and SVM classifier.

Predicted	Actual		
	Gender	Females (%)	Males (%)
CompEn	Females	100	0
	Males	0	100

## Data Availability

All data included in this study are available from the corresponding author upon request.
